# Salinomycin triggers endoplasmic reticulum stress through ATP2A3 upregulation in PC-3 cells

**DOI:** 10.1186/s12885-019-5590-8

**Published:** 2019-04-25

**Authors:** Yunsheng Zhang, Fang Li, Luogen Liu, Hongtao Jiang, Hua Hu, Xiaobo Du, Xin Ge, Jingsong Cao, Yi Wang

**Affiliations:** 1 Clinical Research Institute, The Second Affiliated Hospital, University of South China; Clinical Research Center For Breast & Thyroid Disease Prevention In Hunan Province, Hengyang, 421001 People’s Republic of China; 2 College of Nursing, Hunan Polytechnic of Environment and Biology, Hengyang, 421005 People’s Republic of China; 3 Clinical Research Institute, The Second Affiliated Hospital, University of South China, Hengyang, 421001 People’s Republic of China; 4 Department of Urology, The Second Hospital, University of South China, Hengyang, 421001 People’s Republic of China; 5 Cancer Research Institute, The Second Hospital, University of South China, Hengyang, 421001 People’s Republic of China; 6 Department of Urology, The First People’s Hospital Yueyang, Yueyang, 414000 People’s Republic of China; 7 Clinical Research Institute, The Second Affiliated Hospital, University of South China, Hengyang, 421001 People’s Republic of China; 8 Medical College, Hunan Provincial Key Laboratory for Special Pathogens Prevention and Control, University of South China, Hengyang, 421001 People’s Republic of China; 9 Department of Urology, The Second Affiliated Hospital of Hainan Medical University, Haikou 570102; Clinical Research Institute, The Second Affiliated Hospital, University of South China, Hengyang, 421001 People’s Republic of China

**Keywords:** Salinomycin, ATP2A3, ER stress, Ca^2+^ release, Apoptosis

## Abstract

**Background:**

Salinomycin is a monocarboxylic polyether antibiotic and is a potential chemotherapy drug. Our previous studies showed that salinomycin inhibited cell growth and targeted CSCs in prostate cancer. However, the precise target of salinomycin action is unclear.

**Methods:**

In this work, we analyzed and identified differentially expressed genes (DEGs) after treatment with or without salinomycin using a gene expression microarray in vitro (PC-3 cells) and in vivo (NOD/SCID mice xenograft model generated from implanted PC-3 cells). Western blotting and immunohistochemical staining were used to analyze the expression of ATP2A3 and endoplasmic reticulum (ER) stress biomarkers. Flow cytometry was used to analyze the cell cycle, apoptosis and intracellular Ca^2+^ concentration.

**Results:**

A significantly upregulated gene, ATPase sarcoplasmatic/endoplasmatic reticulum Ca^2+^ transporting 3 (*ATP2A3*), was successfully identified. In subsequent studies, we found that ATP2A3 overexpression could trigger ER stress and exert anti-cancer effects in PC-3 and DU145 cells. ATP2A3 was slightly expressed, but the ER stress biomarkers showed strong staining in prostate cancer tissues. We also found that salinomycin could trigger ER stress, which might be related to ATP2A3-mediated Ca^2+^ release in PC-3 cells. Furthermore, we found that salinomycin-triggered ER stress could promote apoptosis and thus exert anti-cancer effects in prostate cancer cells.

**Conclusion:**

This study demonstrates that ATP2A3 might be one of the potential targets for salinomycin, which can inhibit Ca^2+^ release and trigger ER stress to exert anti-cancer effects.

## Background

Prostate cancer is the second most common malignant cancer in male patients and has high morbidity and mortality [1]. In the past, hormone therapy, surgery and radiation therapy were requirements for advanced prostate cancer; however, since 2004, chemotherapy (docetaxel) has begun to play a significant role [2]. Consequently, finding and studying more specific chemotherapy drugs has important significance for advanced prostate cancer patients. Salinomycin is a monocarboxylic polyether antibiotic isolated from *Streptomyces albus* [3]. In 2009, *Gupta* and colleagues found that salinomycin had nearly 100-fold higher potency against breast cancer stem cells (CSCs) than paclitaxel in a screen of 16,000 compounds [4]. Salinomycin is considered a promising anti-tumor chemotherapy drug, which may reduce the resistance and relapse of cancer by killing cancer cells and CSCs [5].

It has been reported that salinomycin is an ionophore that transports cations (K^+^, Na^+^, Ca^2+^, and Mg^2+^) through cell membranes [6]. Salinomycin can increase intracellular cation concentrations and disrupt the osmotic balance, resulting in apoptosis [7]. In addition, salinomycin is found to inhibit the Wnt/β-catenin signaling pathway and selectively induces apoptosis [8, 9]; reduce the activity of ABC transporters [10]; induce oxidative stress [11], autophagy [12, 13], and anti-angiogenic and anti-tumorigenic activities [14]; inhibit EMT (Epithelial-mesenchymal transition) [15]; and inhibit cancer cell growth [16, 17]. Despite all of this evidence, the molecular mechanism for salinomycin remains elusive, and the precise target of salinomycin action is unclear.

In our previous studies, we found that salinomycin could kill CSCs in lung cancer and inhibit cell growth and target CSCs in prostate cancer [5, 18]. The cytotoxicity of salinomycin to human prostate cancer PC-3 cells was stronger than to nonmalignant prostate cells RWPE-1. Salinomycin induced apoptosis of PC-3 cells by Wnt/β-catenin signaling pathway. Salinomycin, but not paclitaxel, triggered more apoptosis in aldehyde dehydrogenase- (ALDH-) positive PC-3 cells, which were considered as the prostate cancer stem cells, suggesting that salinomycin may be a promising chemotherapeutic to target CSCs [5]. Furthermore, we found that salinomycin-induced autophagy blocks apoptosis via the ATG3/AKT/mTOR signaling axis in prostate cancer PC-3 cells [19]. Salinomycin induced apoptosis and autophagy in PC-3 cells. Interestingly, autophagy inhibition enhanced salinomycin-induced apoptosis. ATG3 was involved in the blockage of apoptosis by autophagy in salinomycin-treated PC-3 cells. ATG3 regulation might occur through the AKT/mTOR signaling axis [19]. However, our previous studies did not address the precise target of salinomycin action.

To investigate the mechanism of salinomycin, a microarray analysis was used to identify DEGs in vitro (PC-3 cells) and in vivo (NOD/SCID mice xenograft model generated from implanted PC-3 cells). ATPase sarcoplasmatic/ endoplasmatic reticulum Ca^2+^ transporting 3 (*ATP2A3*), a significantly upregulated gene, was successfully identified, which encoded one of the Ca^2+^-ATPases. It is known that ATP2A3 is localized in the ER membrane and involves in Ca^2+^ transport [20, 21]. *Griffin* et al. found that the expression of ATP2A3 was downregulated in Jurkat cells, reducing the transport of Ca^2+^ from the cytoplasm into the ER [22]. Other studies found that upregulation of ATP2A3 caused increases in reticular calcium content in the pheochromocytoma cell line PC12 and ultimately resulted in apoptosis [23].

In this study, we found that ATP2A3 might be a potential targets for salinomycin, which inhibits Ca^2+^ release and triggers ER stress. This finding could provide new clues for the mechanism of the salinomycin anti-cancer effects.

## Methods

### Cell culture, drugs and cell survival assay

Human prostate cancer PC-3 and DU145 cells (ATCC, Manassas, VA, USA) were cultured as previously described [5]. Salinomycin (Sigma-Aldrich, St Louis, MO, USA), BAPTA-AM (Selleckchem, Houston, TX, USA) were dissolved in dimethyl sulfoxide (DMSO; Sigma-Aldrich, St Louis, MO, USA). Sodium phenylbutyrate (4-PBA) was dissolved in water.

### Tumorigenic studies in NOD/SCID mice

For tumorigenic studies, PC-3 cells were subcutaneously inoculated into the flanks of NOD/SCID male mice (5 weeks of age; Beijing HFK BioScience Co., Ltd. Beijing China). Mice were housed in a standard laboratory environment (temperature: 24 ± 2 °C; humidity: 50 ± 5%; 12 h day-night cycle) and treated intraperitoneally (i.p.) daily with either DMSO or salinomycin at a dose of 10 mg/kg/day/200 μL (each group was 5). After 3 weeks, the mice were euthanized by carbon dioxide inhalation followed by cervical dislocation. The xenografts were excised and pulverized in liquid nitrogen. Animal studies have approved by the animal ethics committee from South China university.

### Gene expression microarray analysis

Cultured PC-3 cells were treated with 1.0 μM salinomycin or DMSO control for 24 h. Then, total RNA from the abovementioned cells or tumors was extracted with TRIzol reagent (Life Technologies, Inc., Carlsbad, CA, USA) according to the manufacturer’s protocol. Double-stranded cDNA (ds-cDNA) was synthesized from 5 μg of total RNA using a SuperScript ds-cDNA synthesis kit (Life Technologies, Inc., Carlsbad, CA, USA). Human 12 × 135 K Gene Expression Arrays (Roche NimbleGen) were hybridized at 42 °C for 16 to 20 h with 4 μg of Cy3 labeled ds-cDNA in NimbleGen hybridization buffer/hybridization component in a hybridization chamber (Hybridization System-NimbleGen Systems, Inc., Madison, WI, USA).

### Microarray data acquisition and analysis

Slides were scanned at 5 μm/pixel resolution using an Axon GenePix 4000B scanner (Molecular Devices Corporation) piloted by GenePix Pro 6.0 software (Axon). Scanned images (TIFF format) were then imported into NimbleScan software (version 2.5) for grid alignment and expression data analysis. The expression data were normalized through quantile normalization and the Robust Multichip Average (RMA) algorithm included in the NimbleScan software. All gene level files were imported into Agilent GeneSpring GX software (version 11.5.1) for further analysis. Differentially expressed genes were identified through fold Change filtering.

### Quantitative RT-PCR analysis

Quantitative RT-PCR (reverse transcription-polymerase chain reaction) was performed with FastStart Essential DNA Green Master (Roche, Mannheim, Germany). All reactions were performed on the Roche LightCycler 96 Real-Time PCR system (Roche Diagnostics GmbH, Mannheim, Germany). Individual values were normalized to the *GAPDH* loading control. Sequences of gene primers are listed in Table 1. The mRNA expression levels were analyzed using delta cycle threshold (ΔCt) values.

**Table 1:** Primers used for quantitative RT-PCR experiments

Gene name	Forward primer (5′ → 3′)	Reverse primer (5′ → 3′)	Product size (bp)
*MAGEA3*	TCGGTGAGGAGGCAAGGTTC	CGGGAGTGTGGGCAGGAG	123
*ATP2A3*	CTCTGACTTGCCTGGTGGAGA	GGTGAACTCCTTCCGCATCA	122
*NPY1R*	CCTTTGTGAGGTGTTTGTGGG	TGAAGCTAGGAAGAGACGCC	116
*BTBD15*	ACGAGTGCAAAACATGTGGCG	GCCTTTGGAGTGGTACTGTGAA	242
*HSD17B12*	GGAGCAGCGCCTATTAGTGT	CGAAATACGCAGGGCTAGGT	189
*IPF1*	GAATGGCTTTATGGCAGATTA	TGATACTGGATTGGCGTTGT	191
*BGN*	CGGACACACCGGACAGATAG	AAAGGACACATGGCGCTGTA	293
*GAPDH*	GTCTCCTCTGACTTCAACAGCG	ACCACCCTGTTGCTGTAGCCAA	131

### Immunohistochemistry staining

Human prostate cancer tissues and para-carcinoma tissues were obtained from the Second Affiliated Hospital, University of South China with institutional review board approval. Some sections were stained with HE. Immunohistochemistry staining was performed as described previously [24, 25] using ATP2A3 (1:500, GeneTex, San Antonio, TX, USA), BIP and ATF4 antibodies (all from CST, Danvers, MA, USA). Images were captured by a CCD camera (Olympus, Center Valley, PA).

### Western blot analysis

Protein extraction and Western blotting were performed as previously described [26]. The primary antibodies BIP, PERK, ATF4, eIF2a, CHOP, Caspase 12, p-PERK, p-eIF2a, p-CaMK-II (all from CST, Danvers, MA, USA), CaMK-II (Bioworld Technology, Inc., Minneapolis, MN, USA) and ATP2A3 (GeneTex, San Antonio, TX, USA) were used to detect the ER stress. PARP, cleaved PARP antibodies (all from CST, Danvers, MA, USA) were used to detect apoptosis. The β-actin antibody (CST, Danvers, MA, USA) was used as an internal control.

### Transmission electron microscopy

For electron microscopy, PC-3 cells were plated at a density of 10^6^ cells in 100 mm cell culture dishes. The cells were treated with salinomycin for 24 h. Subsequently, the cells were harvested, washed in PBS, and fixed in 2.5% glutaraldehyde/0.2 M phosphate buffer solution (pH 7.4) at 4 °C. Finally, cells were detected by transmission electron microscopy (Servicebio Co., Ltd. Wuhan, China).

### Immunofluorescence staining

Immunofluorescence staining was performed after salinomycin treatment, as previously described [27]. BIP (1:200, Abcam, Cambridge, MA, USA) and CHOP (1:200, CST, Danvers, MA, USA) antibodies were used in this experiment. Secondary antibodies conjugated with Alexa Fluor-647 (Abcam, Cambridge, MA, USA) and Alexa Fluor-488 (Abcam, Cambridge, MA, USA) were used. The fluorophore-labeled cells were examined and analyzed by laser scanning confocal microscopy (Olympus, Tokyo, Japan).

### Detection of [Ca^2+^]_i_ by Fluo-3/AM

Intracellular Ca^2+^ release was detected using the fluorescent probe Fluo-3/AM (Beyotime Biotechnology Co., Haimen, China). For salinomycin treatment, PC-3 and DU145 cells were incubated with Fluo-3/AM stock solution (0.5–5 μM) at 37 °C in the dark for 10 min following three washes with PBS. Samples were analyzed by a FACS-Calibur (BD Biosciences, San Jose, CA, USA), and fluo-3 was detected using a 530/30 nm filter. The arithmetic mean of fluo-3 fluorescence intensity was expressed as [Ca^2+^]_i._ Images of these cells were also captured using an inverted fluorescence microscope (Carl Zeiss, Jena, Germany) to observe the green fluorescence. The results were averaged from three independent experiments.

### Plasmid construction and cell transfection

To construct recombinant ATP2A3 plasmids, the ORF of *ATP2A3* was amplified by PCR and subcloned into the pCDH cDNA cloning lentivector (Cat#CD513B-1; SBI, Mountain View, CA) using the following primers:5′-CCCAAGCTTATGGAGGCGGCGCATCTG-3′ (forward, Hind III included) and 5′-CCGCTCGAGCTTCTGGCTCATTTCGTGC-3′ (reverse, Xho I included). All constructs were verified by sequencing (Sanggon Biotech Co., Ltd., Shanghai, China). The pDsRed2-ER plasmid was purchased from Clontech (Palo Alto, CA, USA). Cell transfection was performed with TurboFect™ in vitro Transfection Reagent (Fermentas, Glen Burnie, MD, USA) according to the manufacturer’s instructions.

### Small interfering RNA knockdown

Small interfering RNA (siRNA) was used to knockdown ATP2A3 expression in PC-3 cells. ATP2A3-siRNAs and negative control sequences were synthesized by RiboBio Co., Ltd. (Guangzhou, China). The siRNAs were transfected by Lipofectamin 2000 (Invitrogen, Life Technologies, Inc., Carlsbad, CA, USA) according to the manufacturer’s instructions.

### Cell cycle and apoptosis analysis

PC-3 cells were seeded in six-well plates and then transfected with pCDH cDNA-ATP2A3 or empty vector for 24–48 h. For cell cycle analysis, cells were fixed and stained as previously described [26]. For apoptosis analysis, apoptosis and necrosis were evaluated by annexin V-FITC/PI staining as previously described [26]. The samples were analyzed by a FACS-Calibur (BD Biosciences, San Jose, CA, USA).

### Statistical analysis

The results were representative of at least three replicates except where specified and are shown as the mean ± SD. To compare the rates of cell apoptosis, a chi-square test was used. For WB of protein expression, ImageJ was used to quantify the density of each band, and then the significance of the fold change was determined with one-way analysis of variance (ANOVA); the significance of the difference of mean fluorescence between groups was also tested with ANOVA. The LSD t-test was used to compare the groups. All statistical analyses were performed using the SPSS 18.0 software (SPSS Inc., Chicago, IL, USA) for Windows. A *P* value < 0.05 was considered statistically significant.

## Results

### Identification of DEGs induced by salinomycin in vitro and in vivo

Previously, we found that salinomycin inhibited PC-3 cell proliferation and decreased xenograft tumor size [5]. To investigate the mechanism of salinomycin, a microarray analysis was used to identify differentially expressed genes (DEGs) in vitro (PC-3 cells) and in vivo (NOD/SCID mice xenograft model generated from implanted PC-3 cells) (Fig. 1a). Based on the threshold of *P*-value ≤0.001 and fold change ≥2.0, Venn diagrams showed that 150 DEGs were obtained (Fig. 1b). All target values were log-2 base transformed, and then a heatmap was generated for the 150 DEGs (Fig. 1c). The heatmap results showed distinguishable gene expression profiling between samples.

**Fig. 1:** Gene expression changes induced by salinomycin in vitro and in vivo. **a**. Log–log scatter-plot of the microarray results. Plots in region Y represent upregulated genes, while plots in region X represent downregulated genes. **b**. Venn diagram displaying the number of DEGs. **c**. Heatmap representation of genes whose expression is differently regulated by salinomycin in vitro and in vivo. **d**. Chart showing the enriched gene ontology (GO) terms in the category of biological processes for DEGs. **e**. Chart showing the enriched gene ontology (GO) terms in the category of molecular functions for DEGs. **f**. Validation of the expression of DEGs by quantitative RT-PCR. The expression levels of mRNA were analyzed using delta cycle threshold (ΔCt) values

For the identified DEGs, we performed enrichment analysis in GO categories. The results showed that secondary metabolic process (GO:0019748, false discovery rate (FDR) =1E0) and plasma membrane organization (GO:0007009, FDR =1E0) were significantly enriched in the biological processes (Fig. 1d), and G-protein coupled receptor activity (GO:0004930, FDR =1.77E-1) was significantly enriched in molecular functions (Fig. 1e).

The *P*-value ≤0.001 and fold change ≥3.0 thresholds were set to select genes from the 150 DEGs. This search identified 10 genes that fit these criteria (Table. 2). Then, the 10 identified genes were validated by quantitative RT-PCR. Seven gene expression profiles were similar to those revealed by the microarray data. A significantly upregulated gene, *ATP2A3*, which is known to be involved in Ca^2+^ transport [20], was successfully identified (Fig. 1f). Thus, we hypothesized that ATP2A3 may be a potential target for salinomycin in PC-3 cells.

**Table 2:** The fold changes for each of the 10 genes based on the thresholds of *P*-value ≤0.001 and fold change ≥3.0 in vitro and in vivo

Gene name	SEQ_ID	Fold change (In vitro)	Fold change (In vivo)
*ANXA13*	NM_004306	9.130	5.940
*ADHFE1*	BC047492	7.411	3.540
*BGN*	NM_001711	6.800	4.034
*AKR1B10*	NM_020299	6.092	5.596
*MAGEA3*	NM_005362	5.946	6.655
*HGD*	NM_000187	5.711	10.401
*ATP2A3*	NM_005173	5.480	4.399
*IPF1*	NM_000209	4.944	3.138
*LOC441282*	XM_930548	4.292	8.844
*LOC375323*	BC113964	3.980	3.300
*HSD17B12*	NM_016142	3.459	4.380
*BTBD15*	BC030580	−3.249	−5.321
*NPY1R*	BC071720	−15.017	−3.331

### ATP2A3 overexpression triggered ER stress in prostate cancer cells

We validated the microarray and quantitative PCR results by Western blotting in prostate cancer cells. PC-3 or DU145 cells were treated with 0 (vehicle, DMSO), 0.5, 1.0 and 2.0 μM salinomycin for 24 h, and the expression of ATP2A3 was measured by WB. The results showed that ATP2A3 was upregulated by salinomycin treatment, and higher concentrations resulted in higher expression levels. To investigate the time-course of salinomycin-induced ATP2A3 expression, PC-3 or DU145 cells were also treated with 1.0 μM salinomycin for 0, 6, 12 or 24 h. The WB showed that ATP2A3 was progressively induced by salinomycin (Fig. 2a). The data therefore showed that salinomycin upregulates ATP2A3 expression in dose- and time-dependent manners.

**Fig. 2:** ATP2A3 overexpression triggered ER stress. **a**. Salinomycin induced ATP2A3 upregulation in PC-3 and DU145 cells. **b**. Flow cytometry showed that ATP2A3 overexpression induced cell-cycle arrest in PC-3 and DU145 cells. *P < 0.05, vs. empty vector. **c**. Western blotting showed that ATP2A3 overexpression changed cell-cycle regulatory protein expression levels. **d**. Annexin V-FITC/PI staining showed that ATP2A3 overexpression induced PC-3 and DU145 cells apoptosis. *P < 0.05, vs. empty vector. **e**. Western blotting showed that ATP2A3 overexpression induced cleavage of PARP. **f**. ATP2A3 overexpression triggered ER stress in PC-3 and DU145 cells. Western blotting analysis of BIP, CHOP, Caspase 12, ATF4 expression and PERK, eIF2a phosphorylation level. **g**. Immumohistochemical staining showed that ATP2A3 and ER stress biomarkers (BIP and ATF4) expression in prostate cancer and para-carcinoma tissues. Scale bars, 10 μm

To further confirm the role of ATP2A3, we overexpressed ATP2A3 in prostate cancer cells. The data showed that ATP2A3 overexpression arrested the progression of the cell cycle (Fig. 2b) and decreased the protein levels of cyclin D1 and cyclin E1 (Fig. 2c). Furthermore, ATP2A3 overexpression induced apoptosis (Fig. 2d), and triggered PARP cleavage (Fig. 2e). These results suggest that ATP2A3 overexpression can cause cell cycle arrest and induce apoptosis in prostate cancer cells.

It is known that ATP2A3 controls Ca^2+^ transport and that its aberrant expression can cause ER stress [28, 29]. Thus we analyzed the effect of ATP2A3 overexpression on ER stress in prostate cancer. As expected, ATP2A3 overexpression caused the upregulation of ER stress biomarkers (BIP, CHOP, Caspase 12 and ATF4). Furthermore, the phosphorylation levels of PERK and eIF2a also increased significantly (Fig. 2f). These results suggest that ATP2A3 overexpression can trigger ER stress.

Immunohistochemistry staining was used to evaluate the expression of ATP2A3 and ER stress biomarkers (BIP and ATF4) in human prostate cancer and para-carcinoma tissues. The data showed weak ATP2A3 staining, but the ER stress biomarkers were strongly stained in cancer tissues (Fig. 2g). In conclusion, our results suggest that salinomycin can upregulate ATP2A3 expression, which triggers ER stress to exert anti-cancer effects in prostate cancer cells.

### Salinomycin-triggers ER stress in PC-3 cells

We analyzed the effect of salinomycin on ER stress in prostate cancer PC-3 cells. As expected, salinomycin upregulated the expression of BIP, ATF4, CHOP and caspase-12. The phosphorylation levels of PERK and eIF2a also increased significantly (Fig. 3a and b). Furthermore, we measured the protein levels of BIP and CHOP by immunofluorescence staining. Consistent with the Western blotting data, the BIP and CHOP antibody staining signals were stronger after salinomycin treatment than before treatment (Fig. 3c).

**Fig. 3:** Salinomycin triggers ER stress. **a**. Western blotting analyzed BIP, CHOP, Caspase 12 and ATF4 expression, and PERK and eIF2a phosphorylation in PC-3 cells treated with indicated concentration of salinomycin or DMSO as control (CON). **b**. The histogram shows fold protein expression normalized to control (ImageJ quantification of blots density from A. was performed, with three independent replicates.*P < 0.05 vs. control). **c**. The expression of BIP and CHOP in PC-3 cells treated as A. were measured by immunofluorescence. Scale bars, 10 μm. **d**. Representative immunofluorescence images of PC-3 cells transfected with pDsRed-ER and then treated with salinomycin. Scale bars, 10 μm. **e**. Transmission electron microscopy to show salinomycin-treated PC-3 cells. Scale bars, 1 μm

To further confirm that salinomycin-triggers ER stress, we transfected PC-3 cells with the pDsRed2-ER plasmid, which was designed for fluorescent labeling of the endoplasmic reticulum and then treated cells with salinomycin. The results showed that the fluorescent labeling of the endoplasmic reticulum became dim (Fig. 3d). Next, we observed the endoplasmic reticulum by transmission electron microscopy. The results showed that the ER membrane of salinomycin-treated PC-3 cells was dilated (Fig. 3e). Our data suggest that salinomycin can trigger ER stress in PC-3 cells.

### Salinomycin-triggered ER stress might be related to ATP2A3-mediated Ca^2+^ release

Because ATP2A3 re-sequesters cytoplasmic Ca^2+^ to the sarcoplasmatic/ endoplasmatic reticulum store, we determined whether salinomycin influences Ca^2+^ release. PC-3 or DU145 cells were treated with the indicated concentration of salinomycin for 24 h, stained with the calcium indicator Fluo-3 AM and analyzed with flow cytometry. As illustrated in Fig. 4a and b, salinomycin significantly inhibited Ca^2+^ release in prostate cancer cells. Next, we transfected PC-3 cells with siRNA to inhibit ATP2A3 expression. Of the three synthetic siRNAs, ATP2A3#2 and ATP2A3#3 greatly knocked down ATP2A3 expression (Fig. 4c). PC-3 cells transfected with siRNA ATP2A3#2 or ATP2A3#3 for 48 h were further treated with 1.0 μM salinomycin for 24 h; afterward, WB was performed to detect ER stress markers (Fig. 4d), or staining with Fluo-3 AM was performed to detect Ca^2+^ concentration changes (Fig. 4e). The results showed that ATP2A3 silencing weakened salinomycin-triggered ER stress, as salinomycin induced upregulation of BIP and CHOP was constrained in cells transfected with siRNA ATP2A3#2 and ATP2A3#3. Similarly, reduced salinomycin-inhibited Ca^2+^ release was also observed. Our results suggest that salinomycin inhibition of Ca^2+^ release might be related to ATP2A3 in PC-3 cells.

**Fig. 4:** Salinomycin-triggered ER stress might be related to ATP2A3-mediated Ca^2+^ release. **a**. Flow cytometry showed that salinomycin inhibited Ca^2+^ release in PC-3 and DU145 cells. **b**. Images were captured using an inverted fluorescence microscope after salinomycin treatment. Scale bars, 10 μm. **c**. ATP2A3 siRNAs (#1, #2 and #3) were respectively transfected in PC-3 cells for 48 h. Western blotting analyzed ATP2A3 protein expression. **d**. ATP2A3 silencing weakened salinomycin-triggered ER stress in PC-3 cells. **e**. ATP2A3 silencing reduced salinomycin-inhibited Ca^2+^ release in PC-3 cells. **f**. Salinomycin changed CaMK activity. The CaMK-II protein expression level and phosphorylation level (Thr 286) were analyzed by Western blotting. **g**. Western blotting showed that BAPTA-AM (10 μM, an intracellular calcium chelator) weakened salinomycin-triggered ER stress

The calcium/calmodulin kinases (CaMKs) are important mediators of intracellular Ca^2 +^ [30]. Thus, we measured the CaMK-II protein expression level and phosphorylation level (Thr 286) to indirectly ascertain CaMK activity changes [31, 32]. The results showed that salinomycin treatment reduced the protein level of CaMK-II, but the phosphorylation level did not change significantly (Fig. 4f). These data suggest that salinomycin-mediated inhibition of Ca^2+^ release might be related to CaMKs via ubiquitin mediated protein degradation [33], which will be one focus of our future studies.

It has been reported that alterations in Ca^2+^ homeostasis are implicated in ER stress. Thus, we pretreated PC-3 cells with BAPTA-AM (10 μM, an intracellular calcium chelator) to assess whether salinomycin triggers ER stress by releasing Ca^2+^. As expected, the data showed that BAPTA-AM could weaken salinomycin-triggered ER stress (Fig. 4g). Our results suggest that salinomycin-triggered ER stress might be related to ATP2A3-mediated Ca^2+^ release in PC-3 cells.

### Salinomycin triggers ER stress leading to apoptosis

Since ER stress has been shown to play a crucial role in apoptosis [34], we co-treated PC-3 cells with salinomycin and 4-phenylbutyrate (4-PBA, 1 mM, an ER stress antagonist) for 24 h. WB was performed to detect the expression of BIP, CHOP, cleaved caspase3 and cleaved PARP. The data showed that 4-PBA significantly reduced salinomycin-triggered ER stress (Fig. 5a) and hampered caspase3 and PARP cleavage (Fig. 5b). The treated cells were also stained with Annexin V-FITC to detect apoptosis. Flow cytometry showed that 4-PBA also significantly decreased salinomycin-induced apoptosis (Fig. 5c). These results suggest that ER stress can promote salinomycin-triggered apoptosis in PC-3 cells.

**Fig. 5:** Salinomycin triggers ER stress leading to apoptosis. **a**. Western blotting showed that 4-PBA weakened salinomycin-triggered ER stress. **b**. Western blotting showed that 4-PBA weakened salinomycin-induced apoptosis. **c**. Flow cytometry showed that 4-PBA weakened salinomycin-induced apoptosis. **d**. Flow cytometry showed that ATP2A3 silencing weakened salinomycin-induced apoptosis

We also transfected PC-3 cells with siRNA to inhibit ATP2A3 expression. Annexin V-FITC staining illustrated that ATP2A3 silencing could inhibit salinomycin-induced apoptosis (Fig. 5d). In conclusion, our data suggest that ER stress promotes salinomycin-induced apoptosis, which might be related to ATP2A3 in PC-3 cells.

## Discussion

Salinomycin has been shown to exert anti-cancer effects in human prostate cancer as well as in other cancers [35]. However, the molecular mechanism of salinomycin is not completely known. Therefore, a microarray-based approach was used and a significantly upregulated gene, *ATP2A3*, was successfully identified in this study. ATP2A3 is involved in Ca^2+^ transport [20]. Coincidentally, a recent study showed that salinomycin’s action is comparable to that of nigericin (K^+^/H^+^ exchanger) [36]. Therefore, we hypothesized that the anti-cancer effects of salinomycin might be associated with cation transport in prostate cancer cells.

Our results showed that salinomycin upregulated the expression of ATP2A3 in PC-3 and DU145 prostate cancer cells. The *ATP2A3* gene encodes Ca^2+^-ATPase3 from the sarco/endoplasmic reticulum (SERCA3), which is expressed in endothelial and epithelial tissues [37, 38]. We found that ATP2A3 was slightly expressed in human prostate cancer tissues, which suggested that the expression of ATP2A3 might be correlated with prostate tumorigenesis. Thus, we investigated the effects of ATP2A3 in PC-3 and DU145 prostate cancer cells. The results showed that ATP2A3 overexpression inhibited cell cycle progression, induced apoptosis, and markedly triggered ER stress. Consistent with previous reports [12, 39], salinomycin triggered ER stress in prostate cancer PC-3 cells.

ER stress is a physiological response that is caused by internal or external stimuli such as oxidative stress [40], ischemia [41], and Ca^2+^ disorders [20]. ER stress is orchestrated by the unfolded protein response (UPR), and failure to adapt to ER stress results in apoptosis [42]. Transient ER stress could activate UPR and promote cell survival [43]. When ER stress is not mitigated, the UPR triggers apoptosis. The UPR is mediated by at least three major stress sensors: IRE1, ATF6 and PERK [42]. Each stress sensor uses a unique mechanism to promote the activation of a specific transcription factor and the upregulation of a subset of UPR target genes. In this study, we found that ATP2A3 overexpression and salinomycin treatment triggered ER stress by the PERK sensor in PC-3 cells. However, ATP2A3 silencing reduced salinomycin-triggered ER stress. Based on these findings, we postulated that salinomycin-triggered ER stress might be related to ATP2A3 upregulation in PC-3 cells.

ATP2A3 is a fundamental for maintaining intracellular [Ca^2+^] homeostasis by pumping Ca^2+^ into the ER of eukaryotic cells [44]. [Ca^2+^]_i_ is a ubiquitous second messenger that operates with versatility in the regulation of several physiological events, such as apoptosis [45]. Alterations to the Ca^2+^ transport or homeostasis machinery have detrimental effects on survival and health [46]. We found that salinomycin inhibited Ca^2+^ release, thereby resulting in ER stress in PC-3 cells. As expected, ATP2A3 silencing reduced the salinomycin-mediated inhibition of Ca^2+^ release. These results suggest ATP2A3 might be a potential target for salinomycin, which inhibits Ca^2+^ release and triggers ER stress to exert anti-cancer effects. Furthermore, our data suggest that salinomycin-mediated inhibition of Ca^2+^ release might be related to CaMKs via ubiquitin mediated protein degradation [33], which will be one focus of our future studies.

## Conclusions

In this study, we identified DEGs) after salinomycin treatment or no-treatment in vitro and in vivo. We further identified ATP2A3 as a potential target for the molecular mechanism of salinomycin, which might inhibit Ca^2+^ release and trigger ER stress to exert its anti-cancer effects.

## Abbreviations

[Ca^2+^]i: Intracellular Ca^2+^
ATP2A3: ATPase sarcoplasmatic/ endoplasmatic reticulum Ca^2+^ transporting 3
CSCs: Cancer stem cells
DGEs: Differentially expressed genes
EMT: Epithelial-mesenchymal transition
ER stress: Endoplasmic reticulum stress
FDR: False discovery rate
RT-PCR: Reverse transcription-polymerase chain reaction
siRNA: small interfering RNA
UPR: Unfolded protein response
